# Application of the unified method to solve the ion sound and Langmuir waves model

**DOI:** 10.1016/j.heliyon.2022.e10924

**Published:** 2022-10-10

**Authors:** Dulal Chandra Nandi, Mohammad Safi Ullah, Harun-Or- Roshid, M. Zulfikar Ali

**Affiliations:** a Department of Statistics, Comilla University, Cumilla-3506, Bangladesh; b Department of Mathematics, Comilla University, Cumilla-3506, Bangladesh; c Department of Mathematics, Pabna University of Science and Technology, Pabna-6600, Bangladesh; d Department of Mathematics, University of Rajshahi, Rajshahi-6205, Bangladesh

**Keywords:** Unified method, Ion sound and Langmuir waves (ISLW) model, Optical soliton, Beat pattern

## Abstract

We present the unified method and use it to integrate the ion sound and Langmuir waves (ISLW) model to retrieve optical soliton solutions. Some new dynamical optical solitons involving the combo of rational, trigonometric, and hyperbolic function solutions are added in this study. The derived optical soliton solutions display various properties such as beat pattern and oscillation with increasing, decreasing, and simultaneously increasing and decreasing amplitudes. Moreover, kink, dark bell, singular kink, single breather, multiple breathers, dark-, bright-, and dark bright periodic waves are founded. Finally, some dynamical characteristics of the acquired solutions are depicted.

## 1 Introduction

Optical solitons are one of the rising research areas for the development of the telecommunication industry. We cannot imagine the operating of optical fiber, email, internet, mobile phones and many other communications except the idea of a solitary wave [1], [2], [3], [4], [5], [6], [7], [8], [9], [10], [11], [12], [13], [14], [15]. In recent years, nonlocal integrable NLS [16], [17] and mKdV [18], [19] equations have been systematically analyzed through the Hirota bilinear technique [20] and the Riemann-Hilbert algorithm [21]. With the development of the soliton concept, various nonlinear models like the Dullin-Gottwald-Holm model [22], the first integro-differential KP hierarchy model [23], the geophysical Korteweg-de Vries model [24], the Korteweg-de Vries-Burgers model [25], the Jimbo-Miwa model [26], and others [27], [28], [29], [30], [31] are emerging in the telecommunication industry. A well-known model, named as the ion sound and Langmuir waves models, was first presented in 1972 [32] and has since received numerous accolades. This model was extensively employed in various solitary wave propagation including plasma. This model can describe the dynamical behavior of the ion sound wave, which is caused by a high-frequency field for the impact of the ponderomotive force and the Langmuir wave, which is one kind of nonlinear evolution equation [33], [34]. To express soliton solutions of the ISLW model, various integration algorithms such as inverse scattering [35], trial equation scheme [36], Sine-Gordan expansion scheme [37], modified Kudraysov scheme [38], extended direct algebraic mapping method [39], and others [40], [41] have been studied. The fractional ISLW model is studied in ref. [42], [43], and the fractional generalized HSC KdV model is studied in ref. [44]. The first goal of this manuscript is to acquire optical soliton solutions that clarify the physical structures of the governing model by the unified technique [45], [46], [47]. This technique is a generalization of two well-known schemes, known as *tanh*-function, and $G^{\prime }/G$-expansion, shown by Akkagil and Aydemir [45]. In 2021, Ullah and others found the singular solution to the LPD equation [46]. This method was also used to solve the Biswas-Arshed nonlinear structure in 2022 [47]. We affirm that the optical soliton solution of the ISLW model in this method has not been studied yet.

## 2 Governing model

The ISLW model has the following form [33], [34]:

(1) $$iQ_{t}+\frac{1}{2}Q_{xx}-RQ=0,\;R_{tt}-R_{xx}-2{\left(|Q{|}^{2}\right)}_{xx}=0.$$

In Eq. (1), $Qe^{iw_{p}t}$ express the normalized electric field of the Longmuir oscillation, *Q* signifies the electrostatic field excitations, $w_{p}$ is the plasma frequency, and the parameter *R* denotes the normalized density perturbation. In engineering and applied sciences, especially in high-frequency cases, the ISLW model is applicable for the impact of ponderomotive force.

## 3 The ODE structure of the model

Assume the subsequent relation for solving Eq. (1):

(2) $$Q(x,t)=U(\psi )e^{i\delta },\;R(x,t)=V(\psi ),\;\psi =px+gt,\;\delta =kx+wt,$$

in which p,g,k, and *w* are real parameters need to be measured afterward. Combining Eq. (2) and Eq. (1) yields

$$\frac{1}{2}p^{2}U^{\prime \prime }+i(g+pk)U^{\prime }-\frac{1}{2}(2w+k^{2})U-UV=0,$$

(3) $$(g^{2}-p^{2})V^{\prime \prime }-4p^{2}(U^{\prime \;2}+UU^{\prime \prime })=0.$$

Separating imaginary and real parts from the first part of Eq. (3) correspondingly gives

(4) $$i(g+pk)U^{\prime }=0,$$

(5) $$p^{2}U^{\prime \prime }-(2w+k^{2})U-2UV=0.$$

From Eq. (4) we get g=−pk. Integrating the 2nd part of Eq. (3) two times with regard to *ψ*, we have

(6) $$V(\psi )=\frac{2}{k^{2}-1}U^{2}(\psi ),$$

where k≠±1. From Eq. (5) and Eq. (6) we have

(7) $$p^{2}(k^{2}-1)U^{\prime \prime }-(k^{2}-1)(2w+k^{2})U-4U^{3}=0.$$

## 4 Summary of the unified method and its application

Suppose the trial solution of Eq. (7) is

(8) $$U(\psi )=\sum_{i=0}^{N}l_{i}\zeta {\left(\psi \right)}^{i}+\sum_{i=1}^{N}l_{-i}\zeta {\left(\psi \right)}^{-i},$$

(9) $$\zeta^{\prime }(\psi )=\zeta^{2}(\psi )+M.$$

Eq. (9) contains nine types of solutions in three cases:

**Case-01:** Hyperbolic function (when *M* is negative):

(10) $$\zeta (\psi )=\left\{ \begin{array}{c} \frac{\sqrt{-(G^{2}+H^{2})M}-G\sqrt{-M}\cosh(2\sqrt{-M}(\psi +\chi ))}{G\sinh(2\sqrt{-M}(\psi +\chi ))+H},\\ \frac{-\sqrt{-(G^{2}+H^{2})M}-G\sqrt{-M}\cosh(2\sqrt{-M}(\psi +\chi ))}{G\sinh(2\sqrt{-M}(\psi +\chi ))+H},\\ \sqrt{-M}+\frac{2G\sqrt{-M}}{G+\cosh(2\sqrt{-M}(\psi +\chi ))-\sinh(2\sqrt{-M}(\psi +\chi ))},\\ -\sqrt{-M}+\frac{2G\sqrt{-M}}{G+\cosh(2\sqrt{-M}(\psi +\chi ))-\sinh(2\sqrt{-M}(\psi +\chi ))}, \end{array}\right.$$

**Case-02:** Trigonometric function (when *M* is positive):

(11) $$\zeta (\psi )=\left\{ \begin{array}{c} \frac{\sqrt{(G^{2}-H^{2})M}-G\sqrt{M}\cos(2\sqrt{M}(\psi +\chi ))}{G\sin(2\sqrt{M}(\psi +\chi ))+H},\\ \frac{-\sqrt{(G^{2}-H^{2})M}-G\sqrt{M}\cos(2\sqrt{M}(\psi +\chi ))}{G\sin(2\sqrt{M}(\psi +\chi ))+H},\\ i\sqrt{M}+\frac{-2iG\sqrt{M}}{G+\cos(2\sqrt{M}(\psi +\chi ))-i\sin(2\sqrt{M}(\psi +\chi ))},\\ -i\sqrt{M}+\frac{2iG\sqrt{M}}{G+\cos(2\sqrt{M}(\psi +\chi ))-i\sin(2\sqrt{M}(\psi +\chi ))}, \end{array}\right.$$

**Case-03:** Rational function (when M=0)

(12) $$\zeta (\psi )=-\frac{1}{\psi +\chi },$$

when G≠0, *χ*, and *H* are arbitrary parameters.

By balancing principle for $U^{3}$ and $U^{\prime \prime }$ we have N=1. Putting N=1 in Eq. (8) gives

(13) $$U(\psi )=l_{0}+l_{1}\zeta (\psi )+l_{-1}\zeta {\left(\psi \right)}^{-1}.$$

Combining Eq. (9), Eq. (13) and Eq. (7) and doing simple calculation gives the following three solution sets

(14) $$l_{0}=0,\;l_{-1}=0,\;l_{1}=\pm \frac{p}{2}\sqrt{2k^{2}-2},\;m=p^{2}M-\frac{1}{2}k^{2},$$

(15) $$l_{0}=0,\;l_{1}=0,\;l_{-1}=\pm \frac{pM}{2}\sqrt{2k^{2}-2},\;m=p^{2}M-\frac{1}{2}k^{2},$$

(16) $$l_{0}=0,\;l_{1}=\pm \frac{p}{2}\sqrt{2k^{2}-2},\;l_{-1}=\pm \frac{pM}{2}\sqrt{2k^{2}-2},\;m=-\frac{4p^{2}M+k^{2}}{2}.$$

Using Eq. (2), Eq. (6), Eq. (10)–Eq. (12) and Eq. (14) gives the subsequent eighteen exact solutions of Eq. (1).

$$Q_{11}(x,t)=l_{1}(\frac{\sqrt{-(G^{2}+H^{2})M}-G\sqrt{-M}\cosh(2\sqrt{-M}(\psi +\chi ))}{G\sinh(2\sqrt{-M}(\psi +\chi ))+H})e^{i\delta },$$

$$Q_{12}(x,t)=l_{1}(\frac{-\sqrt{-(G^{2}+H^{2})M}-G\sqrt{-M}\cosh(2\sqrt{-M}(\psi +\chi ))}{G\sinh(2\sqrt{-M}(\psi +\chi ))+H})e^{i\delta },$$

$$Q_{13}(x,t)=l_{1}(\sqrt{-M}\;\;+\frac{2G\sqrt{-M}}{G+\cosh(2\sqrt{-M}(\psi +\chi ))-\sinh(2\sqrt{-M}(\psi +\chi ))})e^{i\delta },$$

$$Q_{14}(x,t)=l_{1}(-\sqrt{-M}\;\;+\frac{2G\sqrt{-M}}{G+\cosh(2\sqrt{-M}(\psi +\chi ))-\sinh(2\sqrt{-M}(\psi +\chi ))})e^{i\delta },$$

$$Q_{15}(x,t)=l_{1}(\frac{\sqrt{(G^{2}-H^{2})M}-G\sqrt{M}\cos(2\sqrt{M}(\psi +\chi ))}{G\sin(2\sqrt{M}(\psi +\chi ))+H})e^{i\delta },$$

$$Q_{16}(x,t)=l_{1}(\frac{-\sqrt{(G^{2}-H^{2})M}-G\sqrt{M}\cos(2\sqrt{M}(\psi +\chi ))}{G\sin(2\sqrt{M}(\psi +\chi ))+H})e^{i\delta },$$

$$Q_{17}(x,t)=l_{1}(i\sqrt{M}+\frac{-2iG\sqrt{M}}{G+\cos(2\sqrt{M}(\psi +\chi ))-i\sin(2\sqrt{M}(\psi +\chi ))})e^{i\delta },$$

$$Q_{18}(x,t)=l_{1}(-i\sqrt{M}+\frac{2iG\sqrt{M}}{G+\cos(2\sqrt{M}(\psi +\chi ))-i\sin(2\sqrt{M}(\psi +\chi ))})e^{i\delta },$$

$$Q_{19}(x,t)=-\frac{l_{1}}{\psi +\chi }e^{i\delta },$$

$$R_{11}(x,t)=\frac{l_{1}^{2}}{k^{2}-1}{\left(\frac{\sqrt{-(G^{2}+H^{2})M}-G\sqrt{-M}\cosh(2\sqrt{-M}(\psi +\chi ))}{G\sinh(2\sqrt{-M}(\psi +\chi ))+H}\right)}^{2},$$

$$R_{12}(x,t)=\frac{l_{1}^{2}}{k^{2}-1}{\left(\frac{-\sqrt{-(G^{2}+H^{2})M}-G\sqrt{-M}\cosh(2\sqrt{-M}(\psi +\chi ))}{G\sinh(2\sqrt{-M}(\psi +\chi ))+H}\right)}^{2},$$

$$R_{13}(x,t)=\frac{l_{1}^{2}}{k^{2}-1}(\sqrt{-M}\;{\;+\frac{2G\sqrt{-M}}{G+\cosh(2\sqrt{-M}(\psi +\chi ))-\sinh(2\sqrt{-M}(\psi +\chi ))})}^{2},$$

$$R_{14}(x,t)=\frac{l_{1}^{2}}{k^{2}-1}(-\sqrt{-M}\;{\;+\frac{2G\sqrt{-M}}{G+\cosh(2\sqrt{-M}(\psi +\chi ))-\sinh(2\sqrt{-M}(\psi +\chi ))})}^{2},$$

$$R_{15}(x,t)=\frac{l_{1}^{2}}{k^{2}-1}{\left(\frac{\sqrt{(G^{2}-H^{2})M}-G\sqrt{M}\cos(2\sqrt{M}(\psi +\chi ))}{G\sin(2\sqrt{M}(\psi +\chi ))+H}\right)}^{2},$$

$$R_{16}(x,t)=\frac{l_{1}^{2}}{k^{2}-1}{\left(\frac{-\sqrt{(G^{2}-H^{2})M}-G\sqrt{M}\cos(2\sqrt{M}(\psi +\chi ))}{G\sin(2\sqrt{M}(\psi +\chi ))+H}\right)}^{2},$$

$$R_{17}(x,t)=\frac{l_{1}^{2}}{k^{2}-1}{\left(i\sqrt{M}+\frac{-2iG\sqrt{M}}{G+\cos(2\sqrt{M}(\psi +\chi ))-i\sin(2\sqrt{M}(\psi +\chi ))}\right)}^{2},$$

$$R_{18}(x,t)=\frac{l_{1}^{2}}{k^{2}-1}(-i\sqrt{M}\;{\;+\frac{2iG\sqrt{M}}{G+\cos(2\sqrt{M}(\psi +\chi ))-i\sin(2\sqrt{M}(\psi +\chi ))})}^{2},$$

$$R_{19}(x,t)=\frac{l_{1}^{2}}{k^{2}-1}{\left(\frac{1}{\psi +\chi }\right)}^{2},$$

where ψ=px+gt, δ=kx+mt, $m=p^{2}M-\frac{1}{2}k^{2}$ and $l_{1}=\pm \frac{p}{2}\sqrt{2k^{2}-2}$.

Again, using Eq. (2), Eq. (6), Eq. (10)-Eq. (12) and Eq. (15) offer the following sixteen exact solutions of Eq. (1).

$$Q_{21}(x,t)=l_{-1}{\left(\frac{\sqrt{-(G^{2}+H^{2})M}-G\sqrt{-M}\cosh(2\sqrt{-M}(\psi +\chi ))}{G\sinh(2\sqrt{-M}(\psi +\chi ))+H}\right)}^{-1}e^{i\delta },$$

$$Q_{22}(x,t)=l_{-1}{\left(\frac{-\sqrt{-(G^{2}+H^{2})M}-G\sqrt{-M}\cosh(2\sqrt{-M}(\psi +\chi ))}{G\sinh(2\sqrt{-M}(\psi +\chi ))+H}\right)}^{-1}e^{i\delta },$$

$$Q_{23}(x,t)=l_{-1}(\sqrt{-M}\;{\;+\frac{2G\sqrt{-M}}{G+\cosh(2\sqrt{-M}(\psi +\chi ))-\sinh(2\sqrt{-M}(\psi +\chi ))})}^{-1}e^{i\delta },$$

$$Q_{24}(x,t)=l_{-1}(-\sqrt{-M}\;{\;+\frac{2G\sqrt{-M}}{G+\cosh(2\sqrt{-M}(\psi +\chi ))-\sinh(2\sqrt{-M}(\psi +\chi ))})}^{-1}e^{i\delta },$$

$$Q_{25}(x,t)=l_{-1}{\left(\frac{\sqrt{(G^{2}-H^{2})M}-G\sqrt{M}\cos(2\sqrt{M}(\psi +\chi ))}{G\sin(2\sqrt{M}(\psi +\chi ))+H}\right)}^{-1}e^{i\delta },$$

$$Q_{26}(x,t)=l_{-1}{\left(\frac{-\sqrt{(G^{2}-H^{2})M}-G\sqrt{M}\cos(2\sqrt{M}(\psi +\chi ))}{G\sin(2\sqrt{M}(\psi +\chi ))+H}\right)}^{-1}e^{i\delta },$$

$$Q_{27}(x,t)=l_{-1}(i\sqrt{M}\;{\;+\frac{-2iG\sqrt{M}}{G+\cos(2\sqrt{M}(\psi +\chi ))-i\sin(2\sqrt{M}(\psi +\chi ))})}^{-1}e^{i\delta },$$

$$Q_{28}(x,t)=l_{-1}(-i\sqrt{M}\;{\;+\frac{2iG\sqrt{M}}{G+\cos(2\sqrt{M}(\psi +\chi ))-i\sin(2\sqrt{M}(\psi +\chi ))})}^{-1}e^{i\delta },$$

$$R_{21}(x,t)=\frac{l_{-1}^{2}}{k^{2}-1}{\left(\frac{\sqrt{-(G^{2}+H^{2})M}-G\sqrt{-M}\cosh(2\sqrt{-M}(\psi +\chi ))}{G\sinh(2\sqrt{-M}(\psi +\chi ))+H}\right)}^{-2},$$

$$R_{22}(x,t)=\frac{l_{-1}^{2}}{k^{2}-1}{\left(\frac{-\sqrt{-(G^{2}+H^{2})M}-G\sqrt{-M}\cosh(2\sqrt{-M}(\psi +\chi ))}{G\sinh(2\sqrt{-M}(\psi +\chi ))+H}\right)}^{-2},$$

$$R_{23}(x,t)=\frac{l_{-1}^{2}}{k^{2}-1}(\sqrt{-M}\;{\;+\frac{2G\sqrt{-M}}{G+\cosh(2\sqrt{-M}(\psi +\chi ))-\sinh(2\sqrt{-M}(\psi +\chi ))})}^{-2},$$

$$R_{24}(x,t)=\frac{l_{-1}^{2}}{k^{2}-1}(-\sqrt{-M}\;{\;+\frac{2G\sqrt{-M}}{G+\cosh(2\sqrt{-M}(\psi +\chi ))-\sinh(2\sqrt{-M}(\psi +\chi ))})}^{-2},$$

$$R_{25}(x,t)=\frac{l_{-1}^{2}}{k^{2}-1}{\left(\frac{\sqrt{(G^{2}-H^{2})M}-G\sqrt{M}\cos(2\sqrt{M}(\psi +\chi ))}{G\sin(2\sqrt{M}(\psi +\chi ))+H}\right)}^{-2},$$

$$R_{26}(x,t)=\frac{l_{-1}^{2}}{k^{2}-1}{\left(\frac{-\sqrt{(G^{2}-H^{2})M}-G\sqrt{M}\cos(2\sqrt{M}(\psi +\chi ))}{G\sin(2\sqrt{M}(\psi +\chi ))+H}\right)}^{-2},$$

$$R_{27}(x,t)=\frac{l_{-1}^{2}}{k^{2}-1}(i\sqrt{M}\;{\;+\frac{-2iG\sqrt{M}}{G+\cos(2\sqrt{M}(\psi +\chi ))-i\sin(2\sqrt{M}(\psi +\chi ))})}^{-2},$$

$$R_{28}(x,t)=\frac{l_{-1}^{2}}{k^{2}-1}(-i\sqrt{M}\;{\;+\frac{2iG\sqrt{M}}{G+\cos(2\sqrt{M}(\psi +\chi ))-i\sin(2\sqrt{M}(\psi +\chi ))})}^{-2},$$

where ψ=px+gt, δ=kx+mt, $m=p^{2}M-\frac{1}{2}k^{2}$ and $l_{-1}=\pm \frac{pM}{2}\sqrt{2k^{2}-2}$.

Using Eq. (2), Eq. (6), Eq. (10)-Eq. (12) and Eq. (16) grant the next eighteen exact solutions of Eq. (1).

$$Q_{31}(x,t)\;=[l_{1}(\frac{\sqrt{-(G^{2}+H^{2})M}-G\sqrt{-M}\cosh(2\sqrt{-M}(\psi +\chi ))}{G\sinh(2\sqrt{-M}(\psi +\chi ))+H})\;+l_{-1}{\left(\frac{\sqrt{-(G^{2}+H^{2})M}-G\sqrt{-M}\cosh(2\sqrt{-M}(\psi +\chi ))}{G\sinh(2\sqrt{-M}(\psi +\chi ))+H}\right)}^{-1}]e^{i\delta },$$

$$Q_{32}(x,t)\;=[l_{1}(\frac{-\sqrt{-(G^{2}+H^{2})M}-G\sqrt{-M}\cosh(2\sqrt{-M}(\psi +\chi ))}{G\sinh(2\sqrt{-M}(\psi +\chi ))+H})\;+l_{-1}{\left(\frac{-\sqrt{-(G^{2}+H^{2})M}-G\sqrt{-M}\cosh(2\sqrt{-M}(\psi +\chi ))}{G\sinh(2\sqrt{-M}(\psi +\chi ))+H}\right)}^{-1}]e^{i\delta },$$

$$Q_{33}(x,t)=[l_{1}(\sqrt{-M}\;\;+\frac{2G\sqrt{-M}}{G+\cosh(2\sqrt{-M}(\psi +\chi ))-\sinh(2\sqrt{-M}(\psi +\chi ))})\;+l_{-1}(\sqrt{-M}\;{\;+\frac{2G\sqrt{-M}}{G+\cosh(2\sqrt{-M}(\psi +\chi ))-\sinh(2\sqrt{-M}(\psi +\chi ))})}^{-1}]e^{i\delta },$$

$$Q_{34}(x,t)=[l_{1}(-\sqrt{-M}\;\;+\frac{2G\sqrt{-M}}{G+\cosh(2\sqrt{-M}(\psi +\chi ))-\sinh(2\sqrt{-M}(\psi +\chi ))})\;+l_{-1}(-\sqrt{-M}\;{\;+\frac{2G\sqrt{-M}}{G+\cosh(2\sqrt{-M}(\psi +\chi ))-\sinh(2\sqrt{-M}(\psi +\chi ))})}^{-1}]e^{i\delta },$$

$$Q_{35}(x,t)=[l_{1}(\frac{\sqrt{(G^{2}-H^{2})M}-G\sqrt{M}\cos(2\sqrt{M}(\psi +\chi ))}{G\sin(2\sqrt{M}(\psi +\chi ))+H})\;+l_{-1}{\left(\frac{\sqrt{(G^{2}-H^{2})M}-G\sqrt{M}\cos(2\sqrt{M}(\psi +\chi ))}{G\sin(2\sqrt{M}(\psi +\chi ))+H}\right)}^{-1}]e^{i\delta },$$

$$Q_{36}(x,t)=[l_{1}(\frac{-\sqrt{(G^{2}-H^{2})M}-G\sqrt{M}\cos(2\sqrt{M}(\psi +\chi ))}{G\sin(2\sqrt{M}(\psi +\chi ))+H})\;+l_{-1}{\left(\frac{-\sqrt{(G^{2}-H^{2})M}-G\sqrt{M}\cos(2\sqrt{M}(\psi +\chi ))}{G\sin(2\sqrt{M}(\psi +\chi ))+H}\right)}^{-1}]e^{i\delta },$$

$$Q_{37}(x,t)\;=[l_{1}(i\sqrt{M}+\frac{-2iG\sqrt{M}}{G+\cos(2\sqrt{M}(\psi +\chi ))-i\sin(2\sqrt{M}(\psi +\chi ))})\;+l_{-1}{\left(i\sqrt{M}+\frac{-2iG\sqrt{M}}{G+\cos(2\sqrt{M}(\psi +\chi ))-i\sin(2\sqrt{M}(\psi +\chi ))}\right)}^{-1}]e^{i\delta },$$

$$Q_{38}(x,t)\;=[l_{1}(-i\sqrt{M}+\frac{2iG\sqrt{M}}{G+\cos(2\sqrt{M}(\psi +\chi ))-i\sin(2\sqrt{M}(\psi +\chi ))})\;+l_{-1}{\left(-i\sqrt{M}+\frac{2iG\sqrt{M}}{G+\cos(2\sqrt{M}(\psi +\chi ))-i\sin(2\sqrt{M}(\psi +\chi ))}\right)}^{-1}]e^{i\delta },$$

$$Q_{39}(x,t)=-[\frac{l_{1}}{\psi +\chi }+l_{-1}{\left(\frac{1}{\psi +\chi }\right)}^{-1}]e^{i\delta },$$

$$R_{31}(x,t)\;=[l_{1}^{2}{\left(\frac{\sqrt{-(G^{2}+H^{2})M}-G\sqrt{-M}\cosh(2\sqrt{-M}(\psi +\chi ))}{G\sinh(2\sqrt{-M}(\psi +\chi ))+H}\right)}^{2}\;\;+l_{-1}^{2}{\left(\frac{\sqrt{-(G^{2}+H^{2})M}-G\sqrt{-M}\cosh(2\sqrt{-M}(\psi +\chi ))}{G\sinh(2\sqrt{-M}(\psi +\chi ))+H}\right)}^{-2}]\frac{1}{k^{2}-1},$$

$$R_{32}(x,t)\;=[l_{1}(\frac{-\sqrt{-(G^{2}+H^{2})M}-G\sqrt{-M}\cosh(2\sqrt{-M}(\psi +\chi ))}{G\sinh(2\sqrt{-M}(\psi +\chi ))+H})\;+l_{-1}{\left(\frac{-\sqrt{-(G^{2}+H^{2})M}-G\sqrt{-M}\cosh(2\sqrt{-M}(\psi +\chi ))}{G\sinh(2\sqrt{-M}(\psi +\chi ))+H}\right)}^{-2}]\frac{1}{k^{2}-1},$$

$$R_{33}(x,t)\;=[l_{1}^{2}{\left(\sqrt{-M}+\frac{2G\sqrt{-M}}{G+\cosh(2\sqrt{-M}(\psi +\chi ))-\sinh(2\sqrt{-M}(\psi +\chi ))}\right)}^{2}\;\;+l_{-1}^{2}(\sqrt{-M}\;{\;+\frac{2G\sqrt{-M}}{G+\cosh(2\sqrt{-M}(\psi +\chi ))-\sinh(2\sqrt{-M}(\psi +\chi ))})}^{-2}]\frac{1}{k^{2}-1},$$

$$R_{34}(x,t)\;=[l_{1}^{2}{\left(-\sqrt{-M}+\frac{2G\sqrt{-M}}{G+\cosh(2\sqrt{-M}(\psi +\chi ))-\sinh(2\sqrt{-M}(\psi +\chi ))}\right)}^{2}\;\;+l_{-1}^{2}(-\sqrt{-M}\;{\;+\frac{2G\sqrt{-M}}{G+\cosh(2\sqrt{-M}(\psi +\chi ))-\sinh(2\sqrt{-M}(\psi +\chi ))})}^{-2}]\frac{1}{k^{2}-1},$$

$$R_{35}(x,t)=[l_{1}^{2}{\left(\frac{\sqrt{(G^{2}-H^{2})M}-G\sqrt{M}\cos(2\sqrt{M}(\psi +\chi ))}{G\sin(2\sqrt{M}(\psi +\chi ))+H}\right)}^{2}\;\;+l_{-1}^{2}{\left(\frac{\sqrt{(G^{2}-H^{2})M}-G\sqrt{M}\cos(2\sqrt{M}(\psi +\chi ))}{G\sin(2\sqrt{M}(\psi +\chi ))+H}\right)}^{-2}]\frac{1}{k^{2}-1},$$

$$R_{36}(x,t)=[l_{1}^{2}{\left(\frac{-\sqrt{(G^{2}-H^{2})M}-G\sqrt{M}\cos(2\sqrt{M}(\psi +\chi ))}{G\sin(2\sqrt{M}(\psi +\chi ))+H}\right)}^{2}\;\;+l_{-1}^{2}{\left(\frac{-\sqrt{(G^{2}-H^{2})M}-G\sqrt{M}\cos(2\sqrt{M}(\psi +\chi ))}{G\sin(2\sqrt{M}(\psi +\chi ))+H}\right)}^{-2}]\frac{1}{k^{2}-1},$$

$$R_{37}(x,t)\;=[l_{1}^{2}{\left(i\sqrt{M}+\frac{-2iG\sqrt{M}}{G+\cos(2\sqrt{M}(\psi +\chi ))-i\sin(2\sqrt{M}(\psi +\chi ))}\right)}^{2}\;\;+l_{-1}^{2}{\left(i\sqrt{M}+\frac{-2iG\sqrt{M}}{G+\cos(2\sqrt{M}(\psi +\chi ))-i\sin(2\sqrt{M}(\psi +\chi ))}\right)}^{-2}]\;\times \frac{1}{k^{2}-1},$$

$$R_{38}(x,t)\;=[l_{1}^{2}{\left(-i\sqrt{M}+\frac{2iG\sqrt{M}}{G+\cos(2\sqrt{M}(\psi +\chi ))-i\sin(2\sqrt{M}(\psi +\chi ))}\right)}^{2}\;\;+l_{-1}^{2}{\left(-i\sqrt{M}+\frac{2iG\sqrt{M}}{G+\cos(2\sqrt{M}(\psi +\chi ))-i\sin(2\sqrt{M}(\psi +\chi ))}\right)}^{-2}]\;\times \frac{1}{k^{2}-1},$$

$$R_{39}(x,t)=[l_{1}^{2}{\left(\frac{1}{\psi +\chi }\right)}^{2}+l_{-1}^{2}{\left(\frac{1}{\psi +\chi }\right)}^{-2}]\frac{1}{k^{2}-1},$$

where ψ=px+gt, δ=kx+mt, $m=-\frac{4p^{2}M+k^{2}}{2}$, $l_{1}=\pm \frac{p}{2}\sqrt{2k^{2}-2}$, and $l_{-1}=\pm \frac{pM}{2}\sqrt{2k^{2}-2}$.

## 5 Figure analysis

The solutions $Q_{11},Q_{12},Q_{21},Q_{22},Q_{31}$, and $Q_{32}$ give similar behavior as depicted in Fig. 1 **(a-c)** by $Q_{21}$. The character of this graph changes based on the condition for parameter *x*. We see that Fig. 1 **(a)** displays oscillations with rapidly growing amplitudes at x=−1; Fig. 1 **(b)** illustrates oscillations with rapidly reducing amplitudes, then drops to 0, and then again oscillations with rapidly growing amplitudes at x=−1/7; and Fig. 1 **(c)** exhibits oscillations with rapidly reducing amplitudes at x=1. A combination of rational polynomials and periodic solitons produces periodic waves $Q_{19}$ and $Q_{39}$, as depicted in Fig. 2 **(a-d)** by $Q_{39}$. The combo periodic optical soliton solutions $Q_{13},Q_{23}$, and $Q_{33}$ exhibit similar behavior and can increase or decrease wave amplitudes. Optical communication systems make use of this property extensively. In particular, we depicted the solution $Q_{13}$ in Fig. 3 **(a-c)**. We see that for k>0, the wave amplitude increases with a constant height after a definite time (see Fig. 3 **(a)**); for k=0 (see Fig. 3 **(b)**), it remains the same; and for k>0, it decreases (see Fig. 3 **(c)**). The solutions $Q_{14},Q_{24}$, and $Q_{34}$ represent double periodic optical solutions as depicted in Fig. 4 **(a-d)** by $Q_{14}$. This diagram displays oscillations with rapidly decreasing amplitudes, which diminish to 0 at the origin and then increase rapidly. Moreover, the solutions $Q_{15},Q_{16}$, $Q_{17},Q_{18}$, $Q_{25},Q_{26},Q_{27},Q_{28},Q_{35},Q_{36},Q_{37}$, and $Q_{38}$ also display beat pattern, as shown by the solution $Q_{25}$ in Fig. 5 **(a-f)**. When G=1, the solution represents a singular wave (see Fig. 5 **(a-c)**). When G=2, the solution is not a singular wave (see Fig. 5 **(d-f)**). The solutions $R_{13},R_{23}$ and $R_{33}$ exhibit kink soliton, as pictured by the solution $R_{13}$ in Fig. 6.1 **(a, b)**. $R_{14}$ and $R_{34}$ exhibit dark bell soliton solution, as pictured by the solution $R_{14}$ in Fig. 6.2 **(a, b)**. $R_{21}$, $R_{22}$, $R_{31}$, and $R_{32}$ exhibit singular kink soliton, as pictured by the solution $R_{22}$ in Fig. 6.3 **(a, b)**. The solutions $R_{11},R_{12},Q_{19},R_{24}$, and $R_{39}$ exhibit a single breather wave solution as shown in Fig. 7.1 **(a, b)** by the solution $R_{11}$. The solutions $R_{17},R_{18},Q_{27},R_{28},\;R_{37}$, and $R_{38}$ exhibit multiple breather wave solutions as depicted in Fig. 7.2 **(a, b)** by $R_{17}$. The solutions $R_{15},R_{16},Q_{25},R_{26},R_{35}$ and $R_{36}$ exhibit the same solution as plotted by the solution $R_{25}$ in Fig. 8 **(a-c)**. This solution represents a dark periodic wave if $G^{2}<H^{2}$ (see Fig. 8 **(a)**), a dark-bright periodic wave if G=±H (see Fig. 8 **(b)**), and a bright periodic wave if $G^{2}>H^{2}$ (see Fig. 8 **(c)**). We can say that the results acquired for the ISLW model in the unified approach are unprecedented and newest.

**Figure 1:** Shape of wave solution *Q*_21_ for *p* = 7, *k* = 2/7, *M* = −1/2, *G* = 1.5, *H* = 1, *χ* = 1, *l*_0_ = *l*_1_ = 0: (a) at *x* = −1, (b) *x* = −1/7, (c) at *x* = 1.

**Figure 2:** Outlook of wave solution *Q*_39_ for *p* = 5, *k* = 4, *M* = 0, *G* = 4, *H* = 1, *χ* = 1, *l*_0_ = 0: (a, c) cubic wave form, (b, d) planner wave form.

**Figure 3:** Plot of wave solution *Q*_13_ for *p* = 10, *M* = −1, *G* = 1, *H* = 1, *χ* = 1, *l*_0_ = *l*_−1_ = 0 at *x* = 0.

**Figure 4:** Profile of solution *Q*_14_ for *p* = 10, *k* = −0.1, *M* = −0.5, *G* = *H* = *χ* = 1, *l*_0_ = *l*_−1_ = 0: (a, c) cubic wave form, (b, d) planner wave form.

**Figure 5:** Shape of *Q*_25_ for *p* = 5, *k* = −1/5, *M* = 2, *H* = *χ* = 1, *l*_0_ = *l*_1_ = 0: (a-c) at *G* = 1, (d-f) at *G* = 2 (a, d) 3D view, (b, e) 2D view, and (c, f) absolute value view.

**Figure 6.1:** Outlook of *R*_13_ for *p* = 1,*k* = 2, *M* = −0.5, *G* = 4, *H* = *χ* = 1, *l*_0_ = *l*_−1_ = 0: (a) 3D surface, (b) 2D surface.

**Figure 6.2:** Outlook of *R*_14_ for *p* = 1, *k* = −1/10, *M* = −1/2, *G* = *H* = *χ* = 1, *l*_0_ = *l*_−1_ = 0: (a) 3D surface, (b) 2D surface.

**Figure 6.3:** Outlook of *R*_22_ for *p* = 2, *k* = −.5, *M* = −.2, *G* = 3, *H* = *χ* = 1, *l*_0_ = *l*_1_ = 0: (a) 3D surface, (b) 2D surface.

**Figure 7.1:** Graphics of *R*_11_ for *p* = 5, *k* = −1/2, *M* = −1, *G* = 4, *H* = *χ* = 1, *l*_0_ = *l*_−1_ = 0: (a) 3D view, (b) 2D view.

**Figure 7.2:** Graphics of *R*_17_ for *p* = 1, *k* = −3, *M* = 2, *G* = *H* = *χ* = 1, *l*_0_ = *l*_−1_ = 0: (a) 3D shape, (b) 2D shape.

**Figure 8:** Wave pattern of wave solution *R*_25_ for *p* = 1, *k* = −1/3, *M* = 1/2, *χ* = 1, *l*_0_ = *l*_1_ = 0: (a) dark periodic wave at *G* = 2, *H* = 3, (b) dark-bright periodic wave at *G* = *H* = 3, and (c) bright periodic wave at *G* = 4, *H* = 3.

## 6 Conclusion

This paper has presented the unified method to integrate the ISLW model to retrieve optical solitons that can be used in birefringent fibers. Fig. 2 illustrates periodic waves whose amplitudes increase and decrease. The derived optical soliton solutions exhibit some dynamics as beat pattern, oscillation together increasing, decreasing, and jointly increasing-decreasing amplitudes as shown in Figure 1, Figure 3, Figure 4, Figure 5. Kink, dark bell, and singular kink waves are shown in **Fig. 6**. Single breather and multiple breather waves are shown in **Fig. 7**. Moreover, dark, dark-bright, and bright solitons are shown in Fig. 8. In mathematics and engineering, the mentioned technique is an elegant algorithm for finding optical solitons of nonlinear complex models. In addition, applications of fractional differential equations to ISLW models are described in Ref. [42], [43]. In future studies, we need to develop the fractional differential equation of this model by the unified method.

## Declarations

### Author contribution statement

**Dulal Chandra Nandi:** Analyzed and interpreted the data; Contributed reagents, materials, analysis tools or data. **Mohammad Safi Ullah:** Conceived and designed the experiments; Wrote the paper. **Harun-Or-Roshid; M. Zulfikar Ali:** Performed the experiments.

### Funding statement

This research did not receive any specific grant from funding agencies in the public, commercial, or not-for-profit sectors.

### Data availability statement

No data was used for the research described in the article.

### Declaration of interests statement

The authors declare no conflict of interest.

### Additional information

No additional information is available for this paper.
